The article "Trophoblast cell differentiation in the bovine placenta: differentially expressed genes between uninucleate trophoblast cells and trophoblast giant cells are involved in the composition and remodeling of the extracellular matrix and O-glycan biosynthesis" was published in 2020. Journal: BMC Mol Cell Biol.

# Trophoblast cell differentiation in the bovine placenta: differentially expressed genes between uninucleate trophoblast cells and trophoblast giant cells are involved in the composition and remodeling of the extracellular matrix and O-glycan biosynthesis

**DOI:** 10.1186/s12860-020-0246-8

**Published:** 2020-01-17

**Authors:** Marina Polei, Juliane Günther, Dirk Koczan, Rainer Fürbass

**Affiliations:** 1 Institute of Reproductive Biology, Leibniz Institute for Farm Animal Biology (FBN), 18196 Dummerstorf, Germany; 2 Institute for Genome Biology, Leibniz Institute for Farm Animal Biology (FBN), 18196 Dummerstorf, Germany; 3 Institute of Immunology, University of Rostock, 18057 Rostock, Germany

**Keywords:** UTC, TGC, GO analysis, ECM, Cell migration, Signal transduction

## Abstract

**Background:**

In the bovine placenta, intimate fetomaternal contacts are restricted to discrete placentomes. Here, widely branched fetal chorionic villi interdigitate with corresponding maternal caruncular crypts. The fetal trophoblast epithelium covering the chorionic villi consists of approximately 80% uninucleate trophoblast cells (UTCs) and 20% binuclear trophoblast giant cells (TGCs). The weakly invasive TGCs migrate toward the caruncle epithelium and eventually fuse with individual epithelial cells to form short-lived fetomaternal hybrid cells. In this way, molecules of fetal origin are transported across the placental barrier and released into the maternal compartment. The UTC/TGC ratio in the trophoblast remains almost constant because approximately as many new TGCs are produced from UTCs as are consumed by the fusions. The process of developing TGCs from UTCs was insufficiently understood. Therefore, we aimed to detect differentially expressed genes (DEGs) between UTCs and TGCs and identify molecular functions and biological processes regulated by DEGs.

**Results:**

We analyzed gene expression patterns in virtually pure UTC and TGC isolates using gene arrays and detected 3193 DEGs (*p* < 0.05; fold change values < − 1.5 or > 1.5). Of these DEGs, 1711 (53.6%) were upregulated in TGCs and 1482 (46.4%) downregulated. Gene Ontology (GO) analyses revealed that molecular functions and biological processes regulated by DEGs are related to the extracellular matrix (ECM) and its interactions with cellular receptors, cell migration and signal transduction. Furthermore, there was some evidence that O-glycan biosynthesis in TGCs may produce sialylated short-chain O-glycans (Tn antigen, core 1 O-glycans), while the synthesis of other O-glycan core structures required for the formation of complex (i.e., branched and long-chain) O-glycans appears to be decreased in TGCs.

**Conclusion:**

The differentiation of UTCs into TGCs particularly regulates genes that enable trophoblast cells to interact with their environment. Significant differences between UTCs and TGCs in ECM composition indicate reduced anchoring of TGCs in the surrounding matrix, which might contribute to their migration and their weakly invasive interaction with the maternal endometrium. Furthermore, increased expression of sialylated short chain O-glycans by TGCs could facilitate the modulation of maternal immune tolerance.

## Background

The placenta forms the interface between the fetus and mother. Despite specific anatomical and histological differences among species, the basic functions of the placenta are largely the same: anchoring of the fetus in the uterus, supply of nutrients to the fetus, gas exchange and elimination of fetal waste products. In addition, the placental barrier protects the fetus from harmful substances. By inducing local immune tolerance, the placenta prevents the rejection of the fetus by the mother [1].

The bovine placenta is also an important endocrine organ. The trophoblast autonomously produces significant amounts of estrogens which play a role in softening the birth canal before birth and preparing the mammary gland for lactation. Placental estrogens may also act as local regulators of growth and development of the placenta itself. Furthermore, the placenta is a source of pregnancy-specific peptide hormones, namely, placenta lactogen (PL) and prolactin-related protein I (PRP-I), representing the placental counterparts of the pituitary hormone prolactin (PRL). PL regulates reproductive physiological processes in the uterus and mammary gland and further promotes the release of nutrients from the maternal to the fetal compartment. Remarkably, the functions of PRP-I have not been determined to date (reviewed by [2]). The most conspicuous structures of the bovine placenta are the mushroom-shaped placentomes, which are composed of the fetal chorion and the maternal caruncle. The chorion forms widely ramified villi that protrude into corresponding crypts of the caruncles, resulting in a greatly enlarged fetomaternal contact surface [3–5]. The chorionic villi are covered by the trophoblast epithelium consisting of 80% uninucleate trophoblast cells (UTCs) and 20% binuclear trophoblast giant cells (TGCs), which have a rounded shape and are scattered between the UTCs. The UTC/TGC ratio remains almost constant throughout pregnancy until shortly before birth [6]. UTCs show typical epithelial cell features, being attached to the trophoblast basal lamina and exhibiting tight junctions to neighboring UTCs, creating the placental barrier. The apical surface of UTCs facing the caruncular epithelium exhibits microvilli, thereby also enhancing fetomaternal contacts [6, 7]. TGCs are not connected to the trophoblast basal lamina and do not contribute to the apical surface of the trophoblast epithelium. The two nuclei of TGCs are polyploid as a consequence of acytokinetic mitoses [8, 9]. The cytoplasm of TGCs encloses numerous granules containing different kinds of fetal secretory glycoproteins, such as pregnancy-associated glycoproteins (PAGs), PL and PRP-I [6, 10]. TGCs are capable of migrating toward the maternal compartment and traversing the placental barrier. Eventually, TGCs fuse with single caruncular epithelial cells to form short-lived fetomaternal hybrid cells that deliver their cytoplasmic granules into the maternal compartment. After degranulation, hybrid cells become apoptotic and are eventually resorbed by the trophoblast [6]. The resulting loss of TGCs is compensated by new TGCs formed from UTCs by differentiation. During this process, intermediate developmental stages occur that differ in size, level of polyploidy, abundance of cytoplasmic granules and location in the trophoblast epithelium [8, 9]. Because TGCs do not cross the uterine basal membrane and the opposing chorionic and caruncular epithelial layers remain intact, the bovine placenta is classified as synepitheliochorial [6, 7]. Numerous studies have provided profound knowledge on the morphology and histology of the ruminant placenta and its endocrine and other physiological functions. However, our knowledge of the differentiation of UTCs into TGCs at the gene expression level was sparse. Only after the development of a preparative method for the isolation of virtually pure UTCs and TGCs from bovine placentas [11] did a genome-wide gene expression study on trophoblast cell differentiation become feasible.

The aim of this work was to identify differentially expressed genes (DEGs) between UTCs and TGCs and to gain preliminary insights into biological processes, molecular functions and pathways associated with DEGs through gene ontological (GO) analyses.

## Results

### Gene expression profiles of UTCs and TGCs

Although the sorted UTCs and TGCs were virtually pure and appeared to be morphologically sound [11], their natural gene expression patterns may have been distorted during the long preparation procedure. To address this issue, we used qPCR to measure the transcript abundance of the TGC marker genes *RUM1* and *BERV-K1* in the two trophoblast cell populations. The retroviral *RUM1* and *BERV-K1* genes encode placenta-specific membrane glycoproteins, syncytins, which are involved in the fusion of TGCs with caruncle epithelial cells [12]. Indeed, both transcripts were more abundant in TGCs than in UTCs (Fig. 1). Subsequently, we analyzed genome-wide transcripts of UTCs and TGCs in a microarray approach. A hierarchical cluster analysis showed the correct assignment of the microarray expression data sets to the UTC and TGC groups (Fig. 2). We identified 3193 DEGs, 1711 (53.6%) of which were upregulated in TGCs, and 1482 (46.6%) of which were downregulated (Additional file 1: Table S1-A). In this study, we refer to genes as upregulated when their transcripts were more abundant in TGCs than in UTCs. Accordingly, genes whose transcript amounts were lower in TGCs than in UTCs were regarded as downregulated. We evaluated the micorarray measurements with a spot check by reanalyzing 15 transcripts with qPCR and found that both methods provided largely consistent results (Fig. 3; Additional file 1: Table S1-B).

**Fig. 1:** Relative abundance of *RUM1* and *BERV-K1* transcripts in the UTC and TGC isolates. Mean values ± SEM of *n* = 3 independent measurements and the *p*-values from *t*-tests are shown

**Fig. 2:** Hierarchical cluster analysis of the microarray data. Dendrogram of clustering individual samples of UTC and TGC preparations using centered correlation and average linkage. The dendrogram is based on all data as obtained after the GCRMA normalization. The numbers (#2, #3 and #4) refer to the individual animals [11] from which the trophoblast cells originate

**Fig. 3:** Validation of microarray measurements by qPCR. Fold change values compare TGCs vs. UTCs

### KEGG pathways and GO terms associated with DEGs

First, we were interested in identifying KEGG pathways that possibly play significant roles during the differentiation of UTCs into TGCs. To this end, we searched the KEGG database for associations with DEGs using the DAVID functional annotation tool. Our DAVID-compliant DEG list included 2595 genes (DAVID IDs) (Additional file 1: Table S1-C). The significance of the identified KEGG pathways is indicated by a *p*-value, which depends on the number of associated DEGs. KEGG pathways were considered to be highly regulated by DEGs when the *p*-values were < 0.01 and the Benjamini values were < 0.1 (Table 1).

**Table 1:** KEGG pathways associated with DEGs between UTCs and TGCs

KEGG pathway	Count	*p*-value	Benjamini
bta01100:Metabolic pathways	220	3.50E-07	9.98E-05
bta04142:Lysosome	37	3.35E-06	4.77E-04
bta04510:Focal adhesion	52	5.19E-06	4.93E-04
bta05200:Pathways in cancer	83	1.50E-05	0.001070
bta04015:Rap1 signaling pathway	49	1.13E-04	0.006406
bta05205:Proteoglycans in cancer	46	2.43E-04	0.011478
bta04512:ECM-receptor interaction	25	2.55E-04	0.010338
bta00520:Amino sugar and nucleotide sugar metabolism	17	2.66E-04	0.009449
bta04151:PI3K-Akt signaling pathway	68	6.45E-04	0.020212
bta05144:Malaria	17	9.25E-04	0.026019
bta04960:Aldosterone-regulated sodium reabsorption	14	9.90E-04	0.025336
bta04014:Ras signaling pathway	49	0.001085	0.025443
bta00512:Mucin type O-Glycan biosynthesis	12	0.001811	0.038963
bta05143:African trypanosomiasis	13	0.002009	0.040121
bta04925:Aldosterone synthesis and secretion	21	0.002549	0.047336
bta04360:Axon guidance	29	0.002940	0.051092
bta04310:Wnt signaling pathway	31	0.003058	0.050055
bta04070:Phosphatidylinositol signaling system	24	0.003630	0.055954
bta04931:Insulin resistance	26	0.004451	0.064723
bta00051:Fructose and mannose metabolism	11	0.004894	0.067527
bta00670:One carbon pool by folate	8	0.005739	0.075136

The KEGG pathways and the associated DEGs are shown in the Additional file 1: Table S1-D

Furthermore, we attempted to discover biological processes and molecular functions that are relevant for the formation of TGCs from UTCs. To this end, we performed functional annotation clustering, which combines similar GO terms into annotation clusters (ACs) based on the number of shared DEGs. The ranking of the ACs is based on annotation enrichment scores, which result from the individual *p*-values of the GO terms involved. The assumption is that clusters with the highest enrichment scores indicate the most relevant molecular functions and biological processes. The 15 top-ranking ACs are listed in Table 2.

**Table 2:** Annotation clusters (ACs) of DEG-associated GO terms

AC	Enrichment Score	Topic of clustered GO terms
1	9.47	extracellular exosome; extracellular vesicle
2	7.77	membrane microdomain; membrane raft
3	7.02	lipid metabolic process
4	6.65	(regulation of) cell migration, cell motility
5	6.38	regulation of small GTPase mediated signal transduction
6	5.48	ion binding
7	5.37	positive regulation of cellular protein metabolic process
8	4.98	angiogenesis
9	4.81	(regulation of) signal transduction; cell communication
10	4.36	cell-matrix adhesion
11	4.10	carbohydrate metabolic process
12	4.01	cellular response to chemical stimulus
13	3.76	extracellular matrix
14	3.69	phospholipase activity
15	3.64	GTPase regulator activity

The GO terms and associated DEGs are shown in the Additional file 1: Table S1-E

## Discussion

This first genome-wide gene expression study on UTCs and TGCs of bovine trophoblasts was made possible by the availability of virtually pure cell isolates after a FACS-based purification procedure [11]. The aim of this study was to contribute to a deeper understanding of the differentiation processes involved in the formation of TGCs from UTCs in the bovine trophoblast epithelium. By identifying and analyzing DEGs between UTCs and TGCs, we have obtained evidence of molecular functions, biological processes and pathways that are likely to play important roles in the formation of TGCs.

### Evaluation of the integrity of gene expression patterns in UTCs and TGCs

Evidence from the measurements of the TGC marker transcripts *RUM1* and *BERV-K1* indicated that natural gene expression patterns of UTCs and TGCs did not change substantially during the preparative procedure. This conclusion is further supported by the PAG gene expression patterns resulting from the microarray data. Of more than 20 known PAG genes present in the bovine genome, 17 were differentially expressed in UTCs and TGCs (Table 3; Additional file 1: Table S1-A).

**Table 3:** Expression of PAG genes in UTCs and TGCs. Comparison of expression sites revealed by microarray experiments and published data by others

Gene	REFSEQ number	FC	PAG grouping^a^	Main expression site	
				(array data)	(literature)
*PAG2*	NM_176614	− 1.54	ancient	UTCs	TrE^b^;UTC^c,d^
*PAG8*	NM_176619	−3.57	ancient	UTCs	TrE^b^; UTC^d^
*PAG10*	NM_176621	2.99	ancient	TGCs	TrE^b^; TGC^d^
*PAG11*	NM_176623	−2.22	ancient	UTCs	TrE^b^; TGC^c^
*PAG12*	NM_176622	−3.57	ancient	UTCs	TrE^b^
*PAG1*	NM_174411	3.64	modern	TGCs	TGC^b,c^
*PAG3*	NM_001304568	3.59	modern	TGCs	TGC^b^
*PAG4*	NM_176615	1.78	modern	TGCs	TGC^b^
*PAG5*	NM_176616	2.41	modern	TGCs	TGC^b^
*PAG14*	NM_0031304570	3.99	modern	TGCs	TGC^b^
*PAG15*	NM_176624	3.63	modern	TGCs	TGC^b^
*PAG16*	NM_176625	1.77	modern	TGCs	TGC^b^
*PAG17*	NM_176627	1.94	modern	TGCs	TGC^b^
*PAG18*	NM_176626	1.85	modern	TGCs	TGC^b^
*PAG19*	NM_176628	1.68	modern	TGCs	TGC^b^
*PAG20*	NM_176629	3.37	modern	TGCs	TGC^b^
*PAG21*	NM_176630	3.08	modern	TGCs	TGC^b^

Positive and negative fold change (FC) values indicate upregulation and downregulation of genes in TGCs, respectively. TrE: Trophectoderm; ^a^ [13]; ^b^ [14]; ^c^ [15]; ^d^ [16]

Previous in situ hybridization and immunostaining analyses showed a different cellular distribution of ancient and modern PAGs [13] in the trophoblast epithelium, where ancient PAGs were localized mainly in UTCs and in a small number of TGCs, while modern PAGs were restricted to TGCs [14, 16, 17]. In accordance with the published data, the modern PAG genes were all upregulated in TGCs, while the ancient PAG genes *PAG2*, *PAG8* and *PAG12* were downregulated in TGCs. Interestingly, *PAG10* was also upregulated in TGCs, although it is an ancient PAG. However, this observation is consistent with recent results obtained from immunolocalization experiments by Wallace et al. [16]. Only PAG11 localization experiments yielded inconsistent results: in situ hybridization [14] and microarray results indicate that UTCs are PAG11-producing cells, whereas PAG11 immunostaining was restricted to TGCs [15]. In summary, it can be concluded that our UTCs and TGCs were suitable for microarray experiments. In addition, such UTC and TGC isolates should also be useful for future proteome analyses that could not be performed in this study due to the insufficient number of cells.

### DEGs involved in endocrine functions of the bovine placenta

The bovine placenta is capable of producing estrogens independently of the external supply of C19 precursors, as it expresses all enzymes needed to convert cholesterol into estrogens: side chain cleavage enzyme (CYP11A1), steroid 17-alpha-hydroxylase/17,20 lyase (CYP17A1), 3 beta-hydroxysteroid dehydrogenase/Delta 5➔4-isomerase (HSD3B1) and aromatase (CYP19A1) (reviewed by [2]). We searched our microarray data for the expression of the respective transcripts and found that all were downregulated in TGCs (Additional file 1: Table S1-A) with fold-change values of − 4.17 (*CYP11A1*), − 3.85 (*CYP17A1*), − 1.85 (*HSD3B1*) and − 3.85 (*CYP19A1*). The strong downregulation of *CYP11A1* and *CYP17A1* transcripts during TGC development is consistent with previous observations by other groups. Ben David et al. [18] used immunoelectron microscopy and detected CYP11A1-specific signals only in UTCs, and CYP17A1 was immunolocalized only in UTCs [19]. Shortly after UTCs entered the TGC pathway, both enzymes were no longer detectable. The small difference between UTCs and TGCs in *HSD3B1* expression seems to contradict earlier results from in situ hybridization experiments that showed the staining of immature TGCs, while mature TGCs and UTCs were negative [18]. However, because our FACS procedure was designed to collect UTCs and mature TGCs, the proper HSD3B1-expressing cells, namely, the developing TGCs, were likely underrepresented in our TGC isolates. The strong downregulation of *CYP19A1* mRNA in TGCs detected by our measurements contradicted the immunolocalization of the CYP19A1 protein in immature and mature TGCs but not UTCs [19, 20]. In previous experiments we observed a strong decline only in *CYP19A1* transcripts in primary cultures of bovine trophoblast cells, although *CYP19A1* transcripts were clearly detectable in freshly dissociated cells [21]. The cause of the contradictory results has not been determined, but we suspect that *CYP19A1* expression is particularly sensitive to environmental changes during cell isolation.

The GH/PRL hormones regulate numerous physiological processes related to *reproduction* and lactation in many mammalian species, including cattle [22]. The bovine *GH*/*PRL* gene family comprises one *GH* and one *PRL* gene each, both expressed in the pituitary gland, and derivatives of the *PRL* gene (*CSH2*, *PRP*s) expressed in the placenta [2, 23, 24]. The DEGs encoding placenta-expressed GH/PRL representatives were all upregulated in the TGCs (Table 4; Additional file 1: Table S1-A).

**Table 4:** DEGs encoding members of the PRL family of hormones

DEG	Hormone	FC
*CSH2*	chorionic somatomammotropin hormone 2	1.71
*PRL*	prolactin	3.04
*PRP3*	prolactin-related protein 3	3.32
*PRP4*	prolactin-related protein 13	4.18
*PRP6*	prolactin-related protein VI	2.48
*PRP-VII*	prolactin-related protein VII	2.17
*PRP8*	prolactin-related protein VIII	2.90
*PRP14*	prolactin-related protein 14	3.26

*FC* Fold change; positive values indicate higher transcript abundance in TGCs than in UTCs

Notably, our microarray data showed evidence of placental expression of PRL, mainly in the TGCs. This expression has not been observed in cattle to date. However, placental expression of PRL in TGCs has also been immunologically demonstrated in a giraffe [25] and in elephants [26]. Similar to extrapituitary PRL expression in various human tissues, which is regulated by a nonpituitary *PRL* promoter [27, 28], PRL expression in bovine placenta could also use a previously unknown nonpituitary *PRL* promoter. Placenta PRL could exert local functions that differ from the endocrine effects of pituitary PRL.

### Findings from GO analyses of DEGs

The results of GO term enrichment analyses (Tables 1 and 2) indicate that the differentiation of UTCs in TGCs particularly regulates genes that enable trophoblast cells to interact with their environment (GO terms are “ECM receptor interaction”, “mucin-type O-glycan biosynthesis”, “cell-matrix adhesion” and “regulation of small GTPase-mediated signal transduction”) or that probably play a role in the migration of TGCs (GO terms are “regulation of cell migration”, “focal adhesion”). In the following discussion, we will focus in more detail on ECM-receptor interactions and mucin-type O-glycan biosynthesis.

ECM-receptor interactions: The ECM forms the scaffold and the microenvironment for the cellular components of tissues and is subject to continuous remodeling processes. In addition, the ECM provides biochemical and biomechanical signals essential for tissue morphogenesis and differentiation. (reviewed by [29]). The main macromolecular components of the ECM are fibrous proteins, such as collagens and laminins, as well as proteoglycans. Some components of collagen I (ColI), ColVI and laminins are encoded by DEGs (Table 5).

**Table 5:** DEGs associated with the KEGG pathway “ECM receptor interaction”

DEG	Protein	FC
*COL1A1*	collagen, type I, alpha 1	−1.75
*COL1A2*	collagen, type I, alpha 2	−1.75
*COL6A1*	collagen, type VI, alpha 1	−1.59
*LAMA2*	laminin, alpha 2	−1.79
*LAMA3*	laminin, alpha 3	−1.59
*LAMB1*	laminin, beta 1	−2.50
*ITGA1*	integrin, alpha 1	1.55
*ITGA11*	integrin, ITGA11	−1.54
*ITGA2*	integrin, alpha 2	1.86
*ITGA6*	integrin, alpha 6	−1.75
*ITGB4*	integrin, beta 4	−3.13
*ITGB5*	integrin, beta 5	−2.86
*CD36*	CD36 molecule (thrombospondin receptor)	1.61
*CD44*	CD44 molecule	−1.75
*COMP*	cartilage oligomeric matrix protein	3.20
*DAG1*	dystroglycan 1 (dystrophin-associated glycoprotein)	1.61
*HSPG2*	heparan sulfate proteoglycan 2	−1.52
*IBSP*	integrin-binding sialoprotein	−2.08
*RELN*	reelin	2.56
*SDC4*	syndecan 4	−1.67
*SPP1*	secreted phosphoprotein 1 (osteopontin)	−2,00
*SV2B*	synaptic vesicle glycoprotein 2B	1.74
*THBS1*	thrombospondin 1	−1.64
*THBS4*	thrombospondin 4	−2.33

FC: Fold change; positive and negative values indicate higher and lower transcript abundance in TGCs, respectively

ColI consists of α1(I) and α2(I) chains in a stoichiometric ratio of 2:1 [30]. The corresponding genes, *COL1A1* and *COL1A2*, are both downregulated in the TGCs, probably leading to decreased ColI production, as well. ColVI is predominantly present in the basal lamina. ColVI is a heterotrimeric protein consisting of α1(VI), α2(VI) and α3(VI) subunits [31]. ColVI filaments interact with many other ECM components, including ColI and the ColIV network of the basal lamina. In addition, ColVI filaments interact with the cell surface via integrins [31, 32]. ColVI filaments thus establish the biomechanical connection between cells and ECM. In TGCs, *COL6A1*, encoding the α1(VI) subunit, is downregulated. An earlier study in mice showed that the targeted inactivation of *COL6A1* (*COL6A1* ^−/−^) led to a ColVI-null phenotype [33]. Therefore, the production of ColVI heterotrimers in TGCs is likely to be decreased. Laminins are the major noncollageneous component of the basal lamina and play vital roles in cell differentiation, migration and adhesion. Various domains of the laminin subunits enable interactions with other macromolecules, such as the ColIV network, and with plasma membrane receptors, e.g., dystoglycan and integrins [32, 34]. Laminins consist of α, β and γ chains, which in bovines are encoded by five *LAMA* genes, three *LAMB* genes and three *LAMC* genes. *LAMA2*, *LAMA3* and *LAMB1* are downregulated in TGCs (Table 5). Consequently, the formation of laminin heterotrimers with α1, α2 and β1 subunits in TGCs may also be reduced. This reduction would affect 10 of the 15 naturally occurring laminin types, namely, α1/β1/γ1, α2/β1/γ1, α2/β2/γ1, α3/β2/γ1, α3/β2/γ1, α3/β2/γ1, α3/β3/γ2, α3/β1/γ1, α3/β2/γ1, α4/β1/γ1, α5/β1/γ1, α2/β1/γ3 and α3/β2/γ3 [35].

In addition, some integrin-encoding genes were DEGs (Table 5). Integrins are heterodimeric molecules consisting of an α and a β subunit. Both subunits are transmembrane proteins. Integrins mediate cell-cell interactions, anchor cells to the ECM and connect the intracellular actin cytoskeleton to the ECM, thereby mediating both outside-in and inside-out signal transduction. Integrin-mediated cell adhesion plays an important role in controlling cell migration and differentiation [36]. DEG-encoded integrins are constituents of the α1/β1, α2/β1, α6/β1, α11/β1, α6/β4 and αV/β5 integrin receptors [32]. According to the integrin gene expression data, UTCs produce α6/β1, α11/β1, α6/β4 and αV/β5 integrin receptors that are reduced during TGC formation. In contrast, mature TGCs exhibit more α1/β1 and α2/β1 integrins than UTCs. Notably, these integrins are collagen and/or laminin receptors, except for αV/β5 integrin, which binds osteopontin [32]. The results from studies on human placental cytotrophoblasts (CTBs) suggest that the expression of α1/β1 integrin may play a role in the development of the weakly invasive phenotype of TGCs: invasive CTBs also carry α1/β1 integrin receptors on their surface [37], and α1/β1 integrin receptors are necessary for the invasive migration of CTBs [38]. Similar to UTCs, CTB stem cells that are anchored to the basal lamina of the trophoblast epithelium display α6/β4 integrin receptors that disappear when differentiated into invasive CTBs [37, 38]. Integrin switching in CTBs (α6/β4 is downregulated, and α1/β1 is upregulated) is transcriptionally regulated [38]. Immunohistochemical analyses of various ECM proteins and integrin receptors in bovine placentomes showed strong staining of α6 integrin in UTCs and moderate cytoplasmic staining of α2 integrin in TGCs [39], which is consistent with our microarray data. In addition, strong α6 integrin staining along the cytoplasmic membrane of TGCs was detected, which contradicts the observed downregulation of *ITGA6* transcripts in TGCs.

In addition to the ECM proteins and integrin receptors, enzymes involved in ECM remodeling and modification of cell surface or secreted molecules, including heparanase, metalloproteinases (MMPs, ADAMs, ADAMTSs) and tissue inhibitors of metalloproteinases (TIMPs) [40–43], were encoded by DEGs (Table 6).

**Table 6:** DEGs encoding ECM-modifying enzymes/proteinases and TIMPs

DEG	Protein	FC
*ADAM9*	ADAM metallopeptidase domain 9	−1.75
*ADAM28*	ADAM metallopeptidase domain 28	−1.96
*ADAMTS1*	ADAM metallopeptidase with thrombospondin type 1 motif, 1	1.67
*ADAMTS3*	ADAM metallopeptidase with thrombospondin type 1 motif, 3	−1.54
*ADAMTS9*	ADAM metallopeptidase with thrombospondin type 1 motif, 9	1.63
*ADAMTSL1*	ADAMTS-like 1; PUNCTIN	5.23
*HPSE*	heparanase	3.71
*MMP12*	matrix metallopeptidase 12	−1.96
*MMP13*	matrix metallopeptidase 13 (collagenase 3)	−2.04
*TIMP1*	TIMP metallopeptidase inhibitor 1	−1.56
*TIMP2*	TIMP metallopeptidase inhibitor 2	1.75
*TIMP4*	TIMP metallopeptidase inhibitor 4	1.96
*TLL2*	tolloid-like 2	3.59

FC: Fold change; positive and negative values indicate higher and lower abundance of the transcript in TGCs, respectively

Taken together, our data suggest that there are profound differences between UTCs and TGCs regarding their interactions with the surrounding ECM, signal transduction between the ECM and the actin cytoskeleton and downstream processes. The clearly reduced anchoring of TGCs in the surrounding matrix may be related to their migration and weakly invasive phenotype.

Mucin-type O-glycan biosynthesis: Many proteins, whether secreted or bound to cell surfaces, are O-glycosylated [44]. It is therefore remarkable that our microarray data demonstrate significant regulation of the first steps of O-glycan biosynthesis during the formation of TGCs. The underlying DEGs are shown in Table 7.

**Table 7:** DEGs related to O-glycan biosynthesis

DEGs	FC	Enzyme	Products
*GALNT3*	2.06	N-acetylgalactosaminyltransferase 3	TnAg
*GALNT6*	1.89	N-acetylgalactosaminyltransferase 6	TnAg
*GALNT4*	−2.50	N-acetylgalactosaminyltransferase 4	TnAg
*GALNT7*	−2.13	N-acetylgalactosaminyltransferase 7	TnAg
*GALNT10*	−1.69	N-acetylgalactosaminyltransferase 10	TnAg
*C1GALT1*	1.58	N-acetylgalactosamine 3-beta-galactosyltransferase 1	core 1
*ST3GAL1*	3.76	ST3 beta-galactoside alpha-2,3-sialyltransferase 1	sialylated core 1
*GCNT1*	−3.03	glucosaminyl (N-acetyl) transferase 1	core 2
*GCNT3*	−1.52	glucosaminyl (N-acetyl) transferase 3	core 2; core 4
*GCNT4*	−2.50	glucosaminyl (N-acetyl) transferase 4	core 2
*B3GNT6*	−2.94	beta-1,3-N-acetylglucosaminyltransferase 6	core 3

*TnAg* Tn antigen

The products of these first O-glycan biosynthesis steps are basic O-glycan structures, namely, the Tn antigen and four core O-glycans [45] (Fig. 4). The initiating reaction is the coupling of N-acetylgalactosamine (GalNAc) to serine and threonine residues of proteins catalyzed by many isoforms of polypeptide N-acetylgalactosaminyltransferases (GalNTs) (Fig. 4, reaction 1). These GalNT isoforms differ in substrate specificity, compartmentation and expression regulation, and might provide an additional level of regulation for the initiation of O-glycan biosynthesis [46]. The GalNTs fall into two phylogenetically defined groups, which have different substrate preferences: group I enzymes prefer unmodified peptides, while group II enzymes act on modified peptides [46]. Some of the GalNT genes (*GALNT*s) were identified as DEGs in our microarray study (Table 7). Notably, upregulated (*GALNT3* and *GALNT6*) and downregulated genes (*GALNT4*, *GALNT7* and *GALNT10*) belong to different groups, suggesting different targets for O-glycosylation in UTCs and TGCs. The upregulation of *C1GALT1* and *ST3GAL1* in TGCs (Table 7) may lead to an increased production of core 1 and sialylated core 1 O-glycans (Fig. 4, reactions 2 and 6). Sialylated core 1 O-glycans cannot be further extended [45]. In this context, it should be noted that the overexpression of ST3GAL1 is discussed to promote, for instance, tumorigenesis in breast carcinomas [47]. In contrast to the sialylated core 1 O-glycans, the biosynthesis of all other core O-glycans (i.e., cores 2, 3 and 4) is probably downregulated in TGCs (Fig. 4, reactions 3, 4 and 5), as shown by the downregulation of the respective genes (Table 7). Thus, the conversion of UTCs into TGCs is accompanied by a profound structural change in the produced O-glycans: UTCs express all required core structures for complex O-glycans that are shut down during the differentiation process. In contrast, during TGC maturation, short glycans are increasingly synthesized. Due to the numerous biological functions of O-glycans (see [46, 48] for reviews), this might have far-reaching consequences for the cells, for example, through differently modified secreted ECM components or cell surface proteins that are involved in recognition modulation, cell adhesion and communication between cells and their environment. Sialylated glycans often function as self-associated molecular patterns (SAMPs) that attenuate immune defense via interactions with inhibitory siglecs [49]. Thus, TGCs might evade maternal immune defense by increasing the expression of sialylated core 1 O-glycans on the cell surface. In addition to these general aspects of sialic acids, overexpression of ST3GAL1 is specifically known to increase the migration and invasion capacity in ovarian cancer [50]. Based on numerous studies demonstrating a direct link between ST3GAL1 overexpression and tumorigenesis, it is more likely that comparable effects, such as enhanced migration properties, may also take place in TGCs when ST3GAL1 is upregulated.

**Fig. 4:** Schematic representation of structural changes in mucin type O-glycans associated with the differentiation of UTCs into TGCs. Green and red arrows indicate up- and downregulated reactions, respectively. The numbers next to the arrows stand for DEG-encoded enzymes catalyzing the addition of the different sugars (GALNTs, N-acetylgalactosaminyltransferases; C1GALT, core 1 beta1,3-galactosyltransferase; GCNTs, beta1,6-N-acetylglucosaminyltransferases; B3GNT6, beta1,3-N-acetylglucosaminyltransferase 6; ST3GAL4, ST3 beta-galactoside alpha2,3-sialyltransferase 4). More details are given in the text. (GalNAc, N-acetylgalactosamine; Gal, galactose; GlcNAc, N-acetylgucosamine; SIA, sialic acid). (*Modified from* [45])

## Conclusions

From the results of our microarray data, a number of experimentally verifiable hypotheses could be derived:

1. The bovine trophoblast produces PRL, primarily in the TGCs.
2. ECM composition and cell surface receptors differ significantly between UTCs and TGCs, which affects signal transduction and downstream processes.
3. TGCs produce increased amounts of sialylated short-chain O-glycans, while UTCs can form complex, high-molecular-weight O-glycans.

## Materials

### Bovine UTCs and TGCs

Virtually pure UTCs and TGCs were obtained from bovine placentas from days 118 to 130 of gestation in an earlier study [11] with an optimized fluorescence activated cell sorting (FACS) method. Trophoblast cell isolates from three placentas (#2, #3 and #4) provided sufficient amounts of total RNA for the microarray analysis of this study.

### RNA preparation, cRNA production and labeling, and microarray hybridization

Total RNA for the microarray analysis was extracted from UTCs and TGCs with the NucleoSpin RNA II Kit as described by the manufacturer (Macherey-Nagel, Düren, Germany). RNA was quantified in a NanoDrop 1000 spectrophotometer (PeqLab, Erlangen, Germany) and RNA quality was assessed in a 2100 Bioanalyzer instrument using the RNA 6000 Pico Kit and 2100 Expert Software (Agilent Technologies, Santa Clara, CA, USA). RNA integrity numbers were between 7.2 and 8.8. For RNA processing, labeling and hybridization the respective reagent kits from Affymetrix (Santa Clara, USA) were used as recommended by the supplier. Briefly, 120 ng of total RNA from each cell sample was used for single strand DNA (ssDNA) generation using the Ambion WT (whole transcript) Expression Kit (Thermo Fisher Scientific, Waltham, MA, USA). Fragmentation and labeling were performed using the Affymetrix Gene Chip WT Terminal Labeling and Hybridization Kit. The enzymatically fragmented and end labeled ssDNAs were hybridized to Affymetrix Bovine Gene 1.0 ST Arrays for 16 h at 45 °C in an Affymetrix Gene Chip Hybridization Oven. The microarrays were scanned at a 0.7-μm resolution with the Affymetrix Gene Chip Scanner 3000 7G. The data sets from the microarray experiments have been submitted to the Gene Expression Omnibus (GEO) database (accession number GSE122474).

### Analysis of microarray data

The microarray data were analyzed with the Biometric Research Branch (BRB) Array Tools version 4.4.1 [http://linus.nci.nih.gov/BRB-ArrayTools.html]. Background correction and normalization of the expression values was performed using the GC Robust Multi-Array Average (GC RMA) algorithm [51]. Per definition, transcripts were considered differentially expressed among UTC and TGC groups if fold-change values were ≤ − 1.5 or ≥ 1.5 and the *p-*value of the univariate *t*-test between values paired according the UTC and TGC preparations was < 0.05. False discovery rates (FDR) were calculated but not used as a cut-off criterion.

The DEGs were subjected to gene ontology (GO) term analyses using Database for Annotation, Visualization and Integrated Discovery (DAVID) 6.8 software [52, 53]. To this end, our DEG list was first converted into a DAVID compliant gene list using the Gene List Manager. The pathway analyses were based on the Kyoto Encyclopedia of Genes and Genomes (KEGG) database.

### Reverse transcription of RNA; PCR and quantitative reverse-transcription PCR (qPCR)

Microarray measurements were validated by qPCR measurements of selected transcripts. To this end, total RNA (100 ng) from the UTCs or TGCs was reverse transcribed in a 25-μl reaction volume using a mixture of random hexameric and oligo dT primers (4 and 2 ng/μl, respectively; Roche, Mannheim, Germany) and M-MLV reverse transcriptase (GeneOn, Ludwigshafen, Germany). Complementary DNA was purified with the High Pure PCR Product Purification Kit (Roche). Standard PCR to test the specificity of the primer pairs was conducted in 25 μl reaction buffer containing cDNA, Fast Start Taq DNA Polymerase (MP Biomedicals, Illkirch, France), dNTPs (Roche) and gene-specific primers (Additional file 1: Table S1-F). The cycling conditions were as follows: preincubation at 94 °C for 5 min followed by 30 cycles of denaturation at 95 °C for 5 min, annealing at 60 °C for 1 min, extension at 70 °C for 2 min, and a final elongation at 70 °C for 5 min. The PCR products were verified by cloning and sequencing. For qPCR, cDNA was amplified in a 12-μl reaction volume with the SensiFast SYBR No-ROX Kit (Bioline, Luckenwalde, Germany) and gene-specific primer pairs. For amplification and quantification of the PCR products a Light-Cycler 480 instrument (Roche) was used with the following cycling conditions: preincubation at 95 °C for 5 min, followed by 40 cycles of denaturation at 95 °C for 20 s, annealing at 60 °C for 15 s, and extension at 72 °C for 15 s, and single point fluorescence acquisition at 75 °C for 10 s to avoid quantifying primer artifacts. The generation of only the expected products was confirmed by melting curve analysis and agarose gel electrophoresis. External standard curves were generated by coamplification of various dilutions of cloned PCR products (5 × 10^− 12^ to 5 × 10^− 16^ g DNA/reaction) with the corresponding primer pairs. Transcript abundance measurements were normalized using the *RPS18* transcript as an internal reference.

Statistical analyses were performed with SigmaPlot 12.0 Statistical Analysis System (Jandel Scientific, San Rafael, California, USA). Significance of differences was assessed using the *t*-test, and *p-*values < 0.05 were considered statistically significant. Pearson’s product moment correlation was used to compare microarray and qPCR data.

## Supplementary information

**Additional file 1: Table S1-A.** List of differentially expressed genes (DEGs) between UTCs and TGCs obtained by analyzing microarray data with the BRB Array Tools. **Table S1-B.** Correlation between the microarray and quantitative reverse transcription PCR measurements. **Table S1-C.** List of DAVID IDs generated from the BRB list of DEGs (Table S1-A) using the DAVID Gene List Manager. **Table S1-D.** KEGG pathways that are involved in the differentiation of UTCs into TGCs and associated DEGs. **Table S1-E.** Annotation clusters of GO terms related to UTC differentiation into TGCs and associated DEGs (enrichment score > 2). **Table S1-F.** Sequences of primers used for PCR and quantitative reverse transcription PCR.

## Data Availability

The data sets from the microarray experiments have been submitted to the Gene Expression Omnibus (GEO) database (accession number GSE122474).
